The article "Identification of the HMMR Gene as a Diagnostic and Prognostic Biomarker in Hepatocellular Carcinoma Based on Integrated Bioinformatics Analysis" was retracted in 2023. Reasons: signs of a paper mill; suspected computer-generated content; unreliable results or conclusions; concerns about the data.

# Identification of the HMMR Gene as a Diagnostic and Prognostic Biomarker in Hepatocellular Carcinoma Based on Integrated Bioinformatics Analysis

**DOI:** 10.1155/2021/5970085

**Published:** 2021-06-15

**Authors:** Honglan Guo, Qinqiao Fan

**Affiliations:** ^1^Department of Gastroenterology, The First People's Hospital of Chenzhou City, Chenzhou 423000, Hunan, China; ^2^Department of Hepatobiliary, The First People's Hospital of Chenzhou City, Chenzhou 423000, Hunan, China

## Abstract

**Background:**

We aimed to investigate the expression of the hyaluronan-mediated motility receptor (HMMR) gene in hepatocellular carcinoma (HCC) and nonneoplastic tissues and to investigate the diagnostic and prognostic value of HMMR.

**Method:**

With the reuse of the publicly available The Cancer Genome Atlas (TCGA) data, 374 HCC patients and 50 nonneoplastic tissues were used to investigate the diagnostic and prognostic values of HMMR genes by receiver operating characteristic (ROC) curve analysis and survival analysis. All patients were divided into low- and high-expression groups based on the median value of HMMR expression level. Univariate and multivariate Cox regression analysis were used to identify prognostic factors. Gene set enrichment analysis (GSEA) was performed to explore the potential mechanism of the HMMR genes involved in HCC. The diagnostic and prognostic values were further validated in an external cohort from the International Cancer Genome Consortium (ICGC).

**Results:**

HMMR mRNA expression was significantly elevated in HCC tissues compared with that in normal tissues from both TCGA and the ICGC cohorts (all *P* values <0.001). Increased HMMR expression was significantly associated with histologic grade, pathological stage, and survival status (all *P* values <0.05). The area under the ROC curve for HMMR expression in HCC and normal tissues was 0.969 (95% CI: 0.948–0.983) in the TCGA cohort and 0.956 (95% CI: 0.932–0.973) in the ICGC cohort. Patients with high HMMR expression had a poor prognosis than patients with low expression group in both cohorts (all *P* < 0.001). Univariate and multivariate analysis also showed that HMMR is an independent predictor factor associated with overall survival in both cohorts (all *P* values <0.001). GSEA showed that genes upregulated in the high-HMMR HCC subgroup were mainly significantly enriched in the cell cycle pathway, pathways in cancer, and P53 signaling pathway.

**Conclusion:**

HMMR is expressed at high levels in HCC. HMMR overexpression may be an unfavorable prognostic factor for HCC.

## 1. Introduction

Hepatocellular carcinoma (HCC), the predominant form of 90% of primary liver cancers, is the sixth most common diagnosed malignancies and the fourth leading cause of cancer-related deaths worldwide in 2018 [1, 2]. Approximately 250,000 new cases and more than 500,000–600,000 deaths occur annually due to HCC [3]. Moreover, the incidence of HCC will continue to grow over the next two decades and to peak around 2030 according to a Surveillance, Epidemiology, and End Results (SEER) registry projects study [4]. Despite the great advances in imaging techniques, surgical resection, percutaneous ablation, radiotherapy, and liver transplantation, the 5-year survival rate of HCC remains less than 20% because of the high postoperative recurrence rate and metastasis [5, 6]. During the pathogenesis and progression of HCC, the expression of numerous genes has been aberrantly changed, including the activation of oncogenes and inactivation of tumor suppressor genes [7, 8]. Therefore, exploring more novel effective biomarkers for early diagnosis and precise prognostic prediction is urgently required.

Hyaluronan-mediated motility receptor (HMMR) gene, also known as CD168 and RHAMM, belongs to a group of hyaladherins and encodes HMMR which is involved in cell motility [9]. HRRM is a hyaluronan-binding protein, which is expressed in various tumors, including breast, gastric, lung, prostate, and colorectal cancer [10–13]. HMMR is often upregulated in many tumors and has subsequently been related to cancer progression [14, 15]. For example, HMMR positivity is strongly associated with the invasion and metastasis of gastric cancer, and the HMMR-positive group had a significantly higher mortality than the HMMR-negative group [16]. As for HCC, HMMR levels were closely correlated with liver malignant progression in mice. However, so far, little is known about the role of HMMR in the diagnosis and prognosis of HCC in human. Therefore, in the present study, we first explored the diagnostic and prognostic significance of HMMR in HCC.

In the present study, we have evaluated the expression of HMMR in HCC, analyzed its association between clinicopathological features, and explored the potential diagnostic and prognostic value of HMMR in patients with HCC. We further validated the results in an external cohort from the ICGC. Finally, gene set enrichment analysis (GSEA) was carried out to obtain further insight into the biological pathways involved in HCC pathogenesis related to the HMMR regulatory mechanism.

## 2. Materials and Methods

### 2.1. Patients' Data

In this study, a TCGA-LIHC cohort consisting of samples of 374 human HCC tissues and 50 nonneoplastic tissues, as well as clinicopathological characteristics of patients, was downloaded from the TCGA (https://portal.gdc.cancer.gov/) database. Among them, 370 patients had both HMMR expression data and corresponding clinical data. We extracted the mRNA expression data of HMMR in the TCGA cohort. The clinical data including age, sex, vascular invasion information, histologic grade, pathological stage, survival status, survival time, and family history of cancer were used for secondary analysis. Next, we merged the expression and clinical data. Finally, 370 patients were included. According to the median value of HMMR expression, all patients were divided into high-expression and low-expression groups.

### 2.2. Gene Set Enrichment Analysis

Differences of the biological process and pathways in transcriptome levels between high- and low-HMMR gene expression were analyzed using GSEA in the TCGA cohort. C2 (c2.cp.kegg.v7.0.symbols.gmt) from the Molecular Signatures Database (MSigDB) was used as the reference gene sets. The HMMR expression level was annotated as high or low phenotype. Gene set permutations were conducted 1000 times for each analysis. A gene set was regarded as significantly enriched if a normal *P* value was less than 0.05.

### 2.3. Statistical Analysis

The relationship between HMMR expression and clinicopathological characteristics was evaluated using the Wilcoxon signed-rank test, Kruskal–Wallis test, and logistic regression. Area under the curve (AUC) values obtained from the receiver operating characteristic (ROC) curve analysis was utilized to assess the diagnostic effectiveness of HMMR in both cohorts. Generally, an AUC value of more than 0.85 is considered to have an excellent predictive value [17]. Kaplan–Meier curves were used to compare the differences in the overall survival. A log-rank test was performed to determine the significance of the difference between the survival curves. We used univariate and multivariate Cox regression to analyze the effect of HMMR expression level, as a continuous variable, on prognosis along with other clinical variables. Only those variables with *P* value ≤ 0.05 in the univariate analysis were adjusted in multivariate analysis. *P* value <0.05 was considered to be statistically significant. All statistical analyses were performed using R software (V.3.5.1, R Foundation for Statistical Computing, Vienna, Austria).

### 2.4. Validation in an External Cohort

Furthermore, 240 HCC mRNA expression and 260 cases of patients with clinical data from the International Cancer Genome Consortium (ICGC) database were further downloaded (https://dcc.icgc.org/, LIRI-JP), among which 202 normal samples were from solid tissues and 240 primary HCC patients were included in this study to further validate the results yielded in the TCGA cohort.

## 3. Results

### 3.1. Association between Clinicopathological Parameters and HMMR Expression

Using mRNA data in TCGA-LIHC, we examined the expression profile of the HMMR gene in HCC tissues and the adjacent normal tissues. In order to determine the association between HMMR expression and clinicopathological variables in patients with HCC, data from the 370 patients with HCC were collected and evaluated by the *χ*^2^ test. As demonstrated in Figures 1(a)–1(g), high HMMR expression was associated with histologic grade (*P* < 0.0001), pathological stage (*P*=0.039), and survival status (*P*=0.00023); however, no significant associations were identified with other clinicopathological factors, including age, sex, vascular invasion, and family history of cancer (all *P* values > 0.05). As for the expression levels of HMMR between HCC and normal tissues, the result indicated that HMMR was significantly upregulated in HCC tissues than in adjacent normal tissues (Figure 2(a), *P* < 0.0001). We further compared 50 pairs of HCC tissues and matched adjacent tissues form the TCGA cohort, and the result revealed that HMMR was obviously overexpressed in HCC tissues than adjacent tissues (Figure 2(b), *P* < 0.0001).

Logistic regression analysis demonstrated that HMMR expression in HCC was closely associated with histologic grade (dds risk [OR] = 2.881 for grade 3 vs. grade 1, 95% CI: 1.497–5.685, *P*=0.0017; OR = 3.789 for grade 4 vs. grade 1, 95% CI: 1.053–15.75, *P*=0.0483), and patients survival status (OR = 1.958 for dead vs. alive, 95% CI: 1.272–3.036, *P*=0.0024) (Table 1).

### 3.2. Diagnostic and Prognostic Value of HMMR Expression in HCC

We further evaluated the prognosis significance of HMMR in HCC patients. Kaplan–Meier analyses revealed that high HMMR expression was significantly associated with poor overall survival (Figure 2(c), *P* < 0.0001). To evaluate the diagnostic value of HMMR expression in HCC, we generated a ROC curve for HMMR expression in 370 HCC patients and 50 nonneoplastic tissues. The AUC was 0.969 (95% CI: 0.94.8–0.983), which showed excellent diagnostic value (Figure 2(d)). Subsequently, a Cox regression analysis was conducted to explore the independent risk factors for overall survival. Univariate analysis revealed that age, sex, pathological stage, and HMMR expression were significantly associated with overall survival (all *P* values <0.05). After adjusting other prognostic variables, the multivariate analysis confirmed that high HMMR expression remained an independent factor of poor overall survival (HR = 1.136, 95% CI = 1.0586–1.2194, *P*=0.00039). All other independent risk variables and their HR along with 95% CI are displayed in Tables 2 and 3.

### 3.3. Validation in the ICGC Cohort

To further confirm the conclusions from the TCGA cohort, we used an external cohort from the ICGC to validate the abovementioned results. We further compared 202 normal samples from solid tissues and 240 primary HCC patients, and the result remained demonstrated that HMMR was obviously overexpressed in HCC tissues than adjacent tissues (Figure 3(a), *P* < 0.0001). High HMMR expression was also significantly associated with unfavorable overall survival revealed by Kaplan–Meier analyses (Figure 3(b), *P* < 0.001). Just as expected, it was found that the HMMR showed excellent diagnostic value with an AUC of 0.956 (95% CI = 0.932–0.973) in Figure 3(c). The univariate analysis indicated that high HMMR expression was associated with poor survival (HR = 1.205, *P* < 0.001), as well as age and pathological stage (All *P* < 0.005, Figure 3(d)). After adjusting for other risk factors, the multivariate analysis results showed that HMMR expression remained an independent prognostic predictor for survival in HCC (HR = 1.225, 95% CI: 1.122–1.338, *P* < 0.001), as well as sex and pathological stage (Figure 3(e)). Therefore, we are confident that HMMR provides sufficient value as a novel diagnostic and prognostic biomarker for HCC.

### 3.4. GSEA Identifies HMMR-Related Signaling Pathways

To identify KEGG pathway enrichment of HMMR expression, GSEA was conducted comparing the high and low HMMR expression dataset. Gene sets related to DNA replication (map03030), the cell cycle pathway (map04110), the mTOR signaling pathway (map04150), pathways in cancer (map05200), and the p53 signaling pathway (map04115) might be most significantly associated with prognosis of HCC (Figure 4).

## 4. Discussion

In the current study, using data from TCGA-LIHC, we found that HMMR was significantly overexpressed in HCC than in nonneoplastic tissues both in the TCGA cohort and the ICGC cohort. High expression of HMMR was associated with poor survival outcomes of HCC patients, and this was in accordance with the finding that HMMR overexpression was significantly associated with overall survival in colorectal cancer and acute myeloid leukemia [18, 19]. Recently, a growing number of evidence suggests that HMMR is overexpressed in solid tumors and hematological malignancies, including prostate cancer, bladder cancer, gastric cancer, breast cancer, and leukemia [19–22], and it is not known whether HMMR contributes to HCC prognosis.

By performing univariate and multivariate analysis, we further demonstrated that elevated HMMR expression was an independent prognostic risk factor of shorter overall survival (HR = 1.136, 95% CI = 1.0586–1.2194, *P*=0.00039). The finding was further confirmed in an external cohort (HR = 1.225, 95% CI: 1.122–1.338, *P* < 0.001). Therefore, based on these findings, we are confident that HMMR expression can serve as a promising prognostic biomarker of poor outcome of HCC. HMMR expression was confirmed to be significantly corrected to survival in gastric cancer, breast cancer, colon cancer, and prostate cancer [14, 16, 20, 23], which suggested that HMMR may independently predict survival carcinomas. Furthermore, HMMR also presented excellent diagnostic value to discriminate HCC patients from normal ones with a high AUC of 0.969 (95% CI: 0.94.8–0.983). Excitingly, the outstanding diagnostic ability was also achieved in the ICGC cohort with an AUC of 0.956 (95% CI = 0.932–0.973).

As the receptor for hyaluronan-mediated motility, HMMR was first described by Turley as a soluble hyaluronan-binding protein released by subconfluent migrating cells [24]. It has shown to be a vital cell division gene product in immortalized cancer cells and involved in cell motility and signaling, as well as oncogenic events [25]. It was established that HMMR binds to hyaluronan and regulates microtubule-associated protein interactions with actin [26]. Overexpressed mRNA of HMMR at various stages of colorectal cancer was associated with cancer progression and contributed to colorectal cancer cell migration and dispersal [27]. These evidences may help to explain the possible contribution of HMMR expression to the poor survival in HHC. GSEA showed that genes upregulated in the high-HMMR subgroup were mainly significantly enriched in DNA replication, the cell cycle pathway, pathways in cancer, and the P53 signaling pathway. This was in accordance with its role in regulating mitotic spindle integrity, cell cycle progression, and expression of genes governing reorganization and degradation of the extracellular matrix [25, 28]. The pathways in cancer, mTOR signaling pathway, and P53 signaling pathway have revealed to be play an important role in HCC, which was further confirmed in the present study [29, 30].

To the best of our knowledge, the present study first identifies HMMR as a useful diagnostic biomarker for HCC, as well as a powerful independent prognosis factor for patients with HCC. However, there were several limitations. First, this study only examined the prognostic value of HMMR and its dysregulation at the mRNA level. Second, this study was based on bioinformatics analysis, and more in vivo and in vitro studies should be performed in the future to elucidate the specific mechanism that high expression of HMMR is associated with unfavorable prognosis in HCC patients.

## 5. Conclusions

In summary, based on the analysis of TCGA and ICGC databases, the current study demonstrates that HMMR expression was significantly elevated in HCC tissues. HMMR expression may be a power diagnostic and independent prognostic factor in HCC.

## Figures and Tables

**Figure 1:** HMMR expression in patients with HCC. HMMR expression was compared between HCC samples and normal samples in the TCGA cohort according to (a) age, (b) gender, (c) histologic grade, (d) pathological stage, (e) family history of cancer, (f) vascular invasion, and (g) survival status.

**Figure 2:** The expression patterns and diagnostic and prognostic value of HMMR in HCC. (a) HMMR was significantly highly expressed in cancer tissues compared to normal tissues (*P* < 0.0001). (b) HMMR was expressed at higher levels in HCC compared to 50 pairs of adjacent tissues (*P* < 0.0001). (c) Impact of FEN1 expression on overall survival in gastric cancer patients in the TCGA cohort. (d) Diagnosis value of HMMR expression in HCC.

**Figure 3:** Validation of the expression differences and diagnostic and prognostic value of HMMR in HCC in the International Cancer Genome Consortium cohort. (a) HMMR was expressed at higher levels in HCC compared to normal solid tissues (*P* < 0.0001). (b) High HMMR expression was associated with an unfavorable overall survival in HCC patients (*P*=0.00024). (c) Diagnosis value of HMMR expression in HCC in the International Cancer Genome Consortium cohort. (d) Univariate analysis and (e) multivariate analysis of the correlation of HMMR expression with overall survival among HCC patients.

**Figure 4:** Enrichment plots from gene set enrichment analysis (GSEA). DNA replication, the cell cycle pathway, the mTOR signaling pathway, pathways in cancer, and the P53 signaling pathway might be closely associated with prognosis of HCC.

**Table 1:** Logistic regression of HMMR expression associated with clinical pathological characteristics.

Clinical characteristics	Total (*N*)	Odds ratio in HMMR expression	95% CI	*P*
TNM stage (III + IV vs. I + II)	346	1.623	1.001–2.653	0.051
Grade classification (G2 vs. G1)	232	1.635	0.879–3.115	0.126
(G3 vs. G1)	176	2.881	1.497–5.685	0.002
(G4 vs. G1)	67	3.789	1.053–15.750	0.048
Age (≥ 65 vs. < 65)	370	0.681	0.447–1.033	0.072
Gender (male vs. female)	370	0.884	0.571–1.365	0.580
Family history of cancer (yes vs. no)	319	0.725	0.455–1.149	0.172
Vascular invasion (yes vs. no)	314	1.326	0.832–2.122	0.235
Survival status (dead vs. alive)	370	1.958	1.272–3.036	0.002

**Table 2:** Univariate analysis of the relationship between clinical variables of HCC patients and their overall survival.

Variables	HR	95% CI	*P*
Age	1.021	1.0024–1.0401	0.027
Sex	0.586	0.3732–0.9232	0.021
TNM stage	1.464	1.1416–1.8792	0.003
HMMR	1.137	1.0653–1.2137	<0.001
Grade	1.221	0.8927–1.6686	0.212
Vascular invasion	1.443	0.9038–2.3047	0.124
Family history	1.417	0.9032–2.2250	0.130

TNM, tumor node metastasis; HMMR: hyaluronan-mediated motility receptor; HR: hazard ratio; CI: confidence interval.

**Table 3:** Multivariate analysis of the relationship between clinical variables of HCC patients and their overall survival.

Variables	HR	95% CI	*P*
Age	1.019	0.9993–1.0398	0.058
Sex	0.756	0.4655–1.2279	0.258
TNM stage	1.366	1.0561–1.7672	0.017
HMMR	1.136	1.0586–1.2194	<0.001

TNM, tumor node metastasis; HMMR: hyaluronan-mediated motility receptor; HR: hazard ratio; CI: confidence interval.

## Data Availability

The datasets used in the present study are available from the TCGA (https://portal.gdc.cancer.gov/repository) database and the International Cancer Genome Consortium (https://dcc.icgc.org/) database.
